# Yunnan Black Tea Flavonoids Can Improve Cognitive Dysfunction in Septic Mice by Activating SIRT1

**DOI:** 10.1155/2021/5775040

**Published:** 2021-10-11

**Authors:** Chao Mai, Li Qiu, Yong Zeng, Yiping He

**Affiliations:** ^1^Department of Emergency, Affiliated Hospital of North Sichuan Medical College, Nanchong 637000, Sichuan, China; ^2^Department of Emergency, The Second Affiliated Hospital of Chongqing Medical University, Chongqing 400010, China; ^3^Department of Hepatobiliary, Thyroid and Mammary Glands, The People's Hospital of Liangping District in Chongqing, Chongqing 405200, China

## Abstract

This study explored the effect and mechanism of Yunnan black tea flavonoids (YBTF) on cognitive dysfunction in septic mice. The mice were induced sepsis, the serum was determined using kits, and the tissue was determined by qPCR assay. The Yunnan black tea flavonoids were checked using HPLC. The test results showed that compared with the model group, YBTF could increase the survival rate of the mice; meanwhile, YBTF could also increase the total distance travelled, number of stands, and number of groomings, as well as the number of times crossing the area in the target quadrant. Detection of nerve cells showed that YBTF could reduce the rate of nerve cell apoptosis caused by sepsis. YBTF also reduced the levels of tumor necrosis factor-*α* (TNF-*α*), interleukin-6 (IL-6), interleukin-1 beta (IL-1*β*), and malondialdehyde (MDA) in the hippocampus of septic mice and increased the activity of superoxide dismutase (SOD) and catalase (CAT) enzymes. YBTF could also upregulate the mRNA expression of SOD1, SOD2, CAT, and forkhead box O1 (FOXO1) and downregulate the mRNA expression of TNF-*α*, IL-1*β*, nuclear factor kappa-B (NF-*κ*B), p53, and SIRT1 in the hippocampus of septic mice. The animal experiment results showed that YBTF could improve the cognitive dysfunction of septic mice. The effect of YBTF was weaker than that of dexamethasone, but it could enhance the improvement effect when used in conjunction with dexamethasone. The component analysis results showed that YBTF contained 9 compounds, including catechin, gallocatechin gallate, rutin, hyperoside, epicatechin gallate, dihydroquercetin, quercetin, myricetin, and sulphuretin. From these results, YBTF could activate SIRT1 through its active compound components to improve the cognitive dysfunction of septic mice.

## 1. Introduction

Sepsis is a systemic inflammation caused by the host's unregulated response to infection, which will cause systemic inflammation network effects, gene polymorphisms, immune dysfunction, abnormal blood coagulation, tissue damage, and the body's abnormal response to different infectious pathogenic microorganisms and their toxins [1]. Abnormal reactions and many other aspects are closely related to the pathophysiological changes of the body's multiple systems and organs [2]. Sepsis and its complications are the main causes of death in ICU patients with a fatality rate of 30%–70% [3]. It has been indicated that sepsis survivors exhibit long-term cognitive impairment, including loss of memory, attention, and overall cognitive function. In addition, 70% of sepsis patients may suffer from central nervous system dysfunction secondary to sepsis [4]. Sepsis increases the risk of neurodegenerative diseases and dementia, reduces the patient's quality of life, and places a large burden on the patient's family.

Since it is impossible to obtain the results of bacterial culture in the early stage, empirical antibiotic treatment is usually provided in the early stage of sepsis. However, this indiscriminate use of antibiotics may lead to antibiotic abuse and antibiotic resistance [5]. As an adrenal cortex hormone drug, dexamethasone has good anti-inflammatory, antiallergic, and antitoxic effects. Dexamethasone is also commonly used in the treatment of sepsis, but it may have side effects, such as mental symptoms, emotional instability, and oedema [6]. Thereby, dexamethasone was employed as a positive control in this study. Although the drugs used to treat sepsis at the presenting stage can play a certain role, they all have side effects to a certain extent. Therefore, it is of a considerable significance to find active substances with few side effects for the treatment and adjuvant treatment of sepsis.

Black tea is a kind of fermented tea that originated in China. This tea was introduced to Britain in the sixteenth century and became popular in Europe [7]. Among these teas, Yunnan black tea, which is produced in Yunnan, China, is an important variety. Black tea can help gastrointestinal function, promote appetite, help with urination, eliminate oedema, and strengthen heart function [8]. Since black tea is a fermented tea, a large number of polyphenols are decomposed during the fermentation process, but flavonoids are present in large quantities [9]. The black tea flavonoids can scavenge-free radicals and resist acidification, thus reducing the incidence of myocardial infarction [10]. Meanwhile, black tea also has good anti-inflammatory and sterilization effects. This tea has a certain effect on bacillary dysentery and food poisoning as well as on wounds and bedsores [11]. Since black tea flavonoids have antioxidant, anti-inflammatory, and bactericidal effects, existing studies have shown that black tea flavonoids have no toxicity or adverse effects, and there is potential to apply them in sepsis interventions and adjuvant therapy. This study performed relevant research based on this rationale and observed the effect of YBTF on improving the cognitive dysfunction of septic mice.

SIRT1 is an important nicotinamide adenine dinucleotide-dependent protein lysine deacetylase, which can regulate the stress response, inflammatory signals, apoptosis, and cell senescence. Studies have shown that SIRT1 is also closely related to sepsis [12]. The improvement of cognitive dysfunction in septic mice by activating SIRT1 has been confirmed [13]. This study also focused on the mechanistic study of YBTF's efficacy on sepsis. Through the establishment of animal models, various experimental methods, including molecular biology, were used to observe the effect of YBTF on improving the cognitive dysfunction of septic mice by activating SIRT1. The mechanism of action of YBTF was analysed based on the results obtained for the components of YBTF.

## 2. Materials and Methods

### 2.1. Extraction of Flavonoids from Yunnan Black Tea

A total of 200 g of Yunnan black tea was weighed, crushed, and added to a 5 L beaker; 4 L of 70% ethanol was added to achieve a ratio of black tea to ethanol of 1 : 20. The beaker was sealed with a plastic film and placed in a waterbath for 3 h at 60°C. The crude YBTF extract was obtained after the beaker was taken out and cooled. Then, the crude extract was slowly poured into a glass column containing FL-3 macroporous resin (Shanghai Yiji Industrial Co., Ltd., Shanghai, China). The filtrate that passed through the resin for the first time was discarded, and it was eluted with 70% ethanol until the resin became colourless. The eluted solution was collected in a beaker, and the eluent was evaporated in a rotary drier to obtain the YBTF extract.

### 2.2. Laboratory Animal Grouping and Handling

One hundred 10-week-old male ICR mice (Kay Biological Technology (Shanghai) Co., Ltd., Shanghai, China) were adaptively fed for 1 week in the experimental animal breeding room with the temperature controlled at 21 ± 2°C, humidity at 55 ± 2%, and a light/dark cycle of 12 h. Free eating and drinking were allowed. Then, 100 mice were randomly divided into a normal group, a model group, a YBTF group, a dexamethasone group, and a YBTF + dexamethasone group, with 20 mice in each group.

Except for the normal group, the other mice were induced to develop sepsis by caecal ligation and puncture [14]. The experimental mice were anaesthetized by intraperitoneal injection of 15 mg/kg ketamine and 7.5 mg/kg xylazine. After disinfection with iodophor, a 2 cm incision was made in the midline of the mouse abdomen to expose the caecum. The stool was dragged to the caecum and ligated with 5/0 acrylic thread and fixed under the connecting rod of the ileocaecal area, with care being taken to not cause an intestinal obstruction. An 18-gauge needle was used to puncture the caecum 10 times, and it was squeezed slightly until a small drop of stool appeared. The caecum was placed in the abdominal cavity again, and the wound was sutured.

The mice in the normal group and the model group were intragastrically and intraperitoneally injected with 0.2 mL of normal saline, respectively; mice in the YBTF group were intragastrically administered YBTF at a concentration of 100 mg/kg daily; mice in the dexamethasone group were given a daily intraperitoneal injection of dexamethasone at a concentration of 1 mg/kg and were intragastrically administered 0.2 mL of normal saline; the mice in the YBTF + dexamethasone group were intraperitoneally injected with YBTF at a concentration of 100 mg/kg and dexamethasone at a concentration of 1 mg/kg daily for one week. The survival of the mice was checked every day, and survival analysis was also performed for 1 week. One week later, the mice were sacrificed by cervical dislocation, and the tissues and blood were removed for later use. The Ethical Committee for Animal Experiments at the Chongqing Medical University approved the study (SYXK(YU) 2018–0003).

### 2.3. Open Field Test

A single mouse was placed in a box with 100 cm long, 100 cm wide, and 50 cm deep. The mouse was observed for 5 min from the time it was placed in the box, the video tracking system was used to record the mouse's movements, the total moving distance of the mouse was calculated, and the number of standing episodes and the number of self-grooming episodes were counted [15].

### 2.4. Morris Water Maze Experiment

The Morris water maze device consists of a black circular pool with a height of 60 cm and a diameter of 150 cm, which is divided into 4 visual quadrants and filled with 24 ± 2°C water. A circular platform with a diameter of 10 cm is placed in the centre of the third quadrant, 2 cm below the water surface. For 4 consecutive days, the mice were put into the pool facing the wall, and each mouse entered from the 4 quadrants in turn in the same order. Mice that failed to find the platform within 60 s were guided and allowed to stay on the platform for 10 s. The time the mice took to find the platform was recorded as the incubation period. On day 5, after removal of the platform, the time the mice spent in the target quadrant and the number of times the mice crossed the target quadrant were recorded [16].

### 2.5. Flow Cytometry

The mouse hippocampus tissue was lysed and quickly made into a 1 : 9 homogenate with 4^o^C normal saline and 5 *μ*L Annexin-VFITC. Then, the mixture was incubated in a darkroom for 15 min and was analysed by flow cytometry for cell apoptosis (AccuriC6, BD Biosciences, San Jose, CA, USA) [17].

### 2.6. ELISA Experiment

The mouse hippocampus tissue was lysed and quickly made into a 1 : 9 homogenate with 4°C normal saline, centrifuged at 3000 r/min for 15 min, the supernatant was collected, and the TNF-*α*, IL-6, and IL-1*β* levels were detected according to the ELISA instructions (Nanjing Jiancheng Bioengineering Institute, Nanjing, China) [18].

### 2.7. Oxidative Stress Analysis

The mouse hippocampus tissue was lysed and quickly made into a 1 : 9 homogenate with 4°C normal saline, and the SOD, CAT enzyme activity, and MDA levels were tested according to the instructions (Nanjing Jiancheng Bioengineering Institute, Nanjing, China) [19].

### 2.8. qPCR Experiment

The mouse hippocampus tissue was collected and made into a homogenate; then, the RNA was extracted from the tissue with TRIzol™ (Invitrogen, Carlsbad, CA, USA) and diluted to 1 *μ*g/*μ*L. Then, 1 *μ*L of the diluted RNA solution was taken, and reverse transcription was performed according to the reverse transcription kit method to obtain a cDNA template (Thermo Fisher Scientific, Waltham, MA, USA). Next, 1 *μ*L of cDNA template was mixed with 10 *μ*L of SYBR Green PCR Master Mix, 1 *μ*L of upstream and downstream primers (Thermo Fisher Scientific, Table 1), 7 *μ*L of sterile distilled water, and reacted at 95°C for 60 s, and then, at 95°C for 40 cycles, each cycle was 15 s; next, the mixture reacted at 55°C for 30 s, 95°C for 30 s, and 55°C for 35 s before the reaction ended (StepOnePlus, Thermo Fisher Scientific). The 2^−ΔΔCt^ method was used to calculate the relative gene expression, and GAPDH was used as an internal reference for expression [20, 21].

### 2.9. HPLC

The 2 mg of the dry standard was accurately weighed, methanol was added to bring the volume to 2 mL, and it was made into a solution with a concentration of 1 mg/mL. Meanwhile, the sample solution was drawn into the sample bottle with a disposable needle and filter membrane with a volume of 0.5–1.0 mL. The constituents of flavonoids in Yunnan Black tea were determined by HPLC (UltiMate3000 HPLC System, Thermo Fisher Scientific), chromatographic conditions included determination with Agilent Z orbaxSB-C_18_ column (5 *μ*m, 4.6 × 250 mm), the column temperature was 30°C, the mobile phase was methanol, acetic acid water, acetonitrile, and pure water, the flow rate was 0.5 mL/min, the detection wavelength was 328 nm, and the injection volume was 10 *μ*L. A standard curve was drawn according to the chromatogram with the concentration of each substance being the abscissa, and the peak area being the ordinate [22], and a linear regression equation was used to get *R*^2^. Then, the content of flavonoids in the sample was calculated according to the obtained peak area of the sample, the peak area of the standard in the mixed standard, the sample concentration, the concentration of the standard in the mixed standard, and the injection volume of the standard in the mixed standard.

### 2.10. Statistical Analysis

The average values were obtained in three parallel experiments, which were analysed by SPSS 23 statistical software, and the values were compared between groups by the one-way analysis of variance method. Significant differences between groups were observed at the *P* < 0.05 level.

## 3. Results

### 3.1. Survival Status of Septic Mice

One week after the induction of sepsis, no death was found in the normal group, but there were 8 deaths in the model group, 3 deaths in the YBTF group, 4 deaths in the dexamethasone group, and 1 death in the YBTF + dexamethasone group (Figure 1). Compared with the model group, both YBTF and dexamethasone could reduce the mortality of septic mice, and the combination of YBTF and dexamethasone achieved the best effect.

### 3.2. Cognitive Impairment in Septic Mice

Compared with the normal group, the total distance travelled (m), the number of standing episodes, the number of self-grooming episodes, the time in the target quadrant, and the number of times the mice crossed the region were significantly reduced in the model group, and the latency time was significantly increased (Figure 2). Compared with the model group, the total distance travelled, the number of standing episodes, the number of self-grooming episodes, the time in the target quadrant, and the number of times the mice crossed the region were significantly increased (*P* < 0.05) in the model group, and the latency time was significantly increased (*P* < 0.05) in the dexamethasone, YBTF, and YBTF + dexamethasone groups. The mice in the YBTF + dexamethasone group showed the lowest degree of cognitive impairment.

### 3.3. Apoptosis of Nerve Cell Apoptosis in Mice

Compared with the normal group, the apoptosis of nerve cells in the model group increased significantly; compared with the model group, the apoptosis nerve cell of YBTF, dexamethasone, and the YBTF + dexamethasone groups was reduced, and there was no difference in the nerve cell apoptosis rate of mice in the YBTF and dexamethasone groups, but YBTF + dexamethasone could greatly reduce the apoptosis of nerve cells in mice (Figure 3).

### 3.4. Inflammation in the Hippocampus of Mice

It could be seen from Figure 4 that the levels of inflammatory cytokines TNF-*α*, IL-6, and IL-1*β* were the highest in the model group and the lowest in the normal group. Dexamethasone, YBTF, and YBTF + dexamethasone could significantly reduce (*P* < 0.05) the levels of TNF-*α*, IL-6, and IL-1*β* in the hippocampus of septic mice. YBTF + dexamethasone showed the best effect, with the levels of TNF-*α*, IL-6, and IL-1*β* being closest to the normal group.

### 3.5. Oxidative Stress Response in the Mouse Hippocampus

From Figure 5, it could be seen that SOD and CAT enzyme activities in the hippocampus of the normal group mice were the strongest, while the MDA level was the lowest; the model group mice showed the opposite trend, with the highest MDA level and the lowest SOD and CAT enzyme activities. Dexamethasone, YBTF, and YBTF + dexamethasone could reduce the SOD, CAT enzyme activities, and MDA levels of the hippocampus of mice to the level of the normal group, while the effect of YBTF + dexamethasone was significantly stronger (*P* < 0.05) than that of YBTF and dexamethasone.

### 3.6. mRNA Expression in the Mouse Hippocampus

It could be seen from Figure 6 that the mRNA expression of SOD1, SOD2, CAT, and FOXO1 in the hippocampus of the septic mice (model group) was significantly lower (*P* < 0.05) than that of the other groups, while the mRNA expression of TNF-*α*, IL-1*β*, NF-*κ*B, p53, and SIRT1 was significantly higher (*P* < 0.05) than in the other groups. Dexamethasone, YBTF, and YBTF + dexamethasone could upregulate the mRNA expression of SOD1, SOD2, and CAT in the hippocampus of septic mice and downregulate the mRNA expression of TNF-*α*, IL-1*β*, NF-*κ*B, and p53. YBTF + dexamethasone showed the strongest effect.

### 3.7. Components of YBTF

Through HPLC analysis, the experimental results showed that YBTF contained 9 compounds, including catechin (145.23 mg/g), gallocatechin gallate (31.34 mg/g), rutin (178.31 mg/g), hyperoside (2.48 mg/g), epicatechin gallate (185.30 mg/g), dihydroquercetin (33.12 mg/g), quercetin (10.10 mg/g), myricetin (61.20 mg/g), and sulphuretin (12.30 mg/g, Figure 7). The contents of catechin, rutin, and epicatechin gallate were relatively high.

## 4. Discussion

Sepsis is a common and potentially fatal systemic disease that often leads to uncontrollable inflammation, tissue damage, and multiple organ failure. Sepsis and its complications are the main causes of death in ICU patients [23]. This study found that the survival rate of sepsis mice was reduced after treatment with YBTF, and it could enhance the efficacy of dexamethasone (Figure 1). Cognitive impairment is one of the multiple organ dysfunctions caused by sepsis, which seriously affects the survival and prognosis of patients with sepsis. In this experiment, an open field test was used to reflect the activity and exploration ability of the mice (Figure 2) [24]. The Morris water maze test reflected their learning and cognitive abilities. It was found that the activity and exploration ability and the learning and cognitive ability of septic mice were both weakened, but YBTF could alleviate this effect. This finding preliminarily showed that YBTF could not only improve cognitive dysfunction in sepsis but also enhance the efficacy of drugs (Figure 2).

Excessive inflammation, oxidative stress, and severe neuronal apoptosis are considered to be the potential mechanisms of sepsis-induced brain damage and cognitive impairment [25]. The hippocampus plays a vital role in learning, memorizing, emotion, endocrine, and visceral activities. This study shows that the apoptosis rate of nerve cells in septic mice increased, which is consistent with previous studies [26]. Meanwhile, this study found that YBTF could attenuate this pathological change (Figure 3). Oxidative stress and inflammatory ions are the most important factors that trigger neuronal apoptosis and necrosis [27]. In sepsis, the occurrence of oxidative stress and the release of proinflammatory cytokines are the main causes of neuronal death [28]. TNF-*α*, IL-6, and IL-1*β* are all important proinflammatory factors, which play an important role in the occurrence and development of sepsis [29]. SOD and CAT are important antioxidant enzymes involved in the process of oxidative stress, and MDA is an important product of oxidative damage [30]. Therefore, reducing oxidative stress and inflammatory stress is an important treatment method for cognitive impairment in sepsis. Studies have confirmed that colistin-induced nephrotoxicity and neurotoxicity can be reduced by reducing oxidative stress, inflammation, and cell apoptosis in animals [31]. The same study also found that YBTF significantly reduced the levels of TNF-*α*, IL-6, IL-1*β*, and MDA (Figure 4) in hippocampal tissues of septic mice and increased SOD and CAT activities (Figure 5), indicating that YBTF could attenuate the inflammation and oxidative stress response of septic mice.

The activation of SIRT1 inhibits apoptosis, oxidation, and inflammatory ions, thereby reducing the multiple organ damage caused by sepsis, including of the lung, kidney, and liver [32]. The neuroprotective effect of SIRT1 has been confirmed in craniocerebral trauma, ischaemic injury, and many neurodegenerative diseases [33]. This study found that YBTF can upregulate the expression of SIRT1, indicating that YBTF may improve the cognitive dysfunction of septic mice by activating SIRT1 (Figure 6).

When SIRT1 is activated, it exerts antiapoptotic, antioxidant, and anti-inflammatory effects. It is closely related to the deacetylation of downstream signalling proteins (such as FOXO1, p53, and NF-*κ*B) mediated by SIRT1 [34]. FOXO1 is regarded as a metabolic and antioxidant regulator, which can promote the synthesis of SOD and CAT, especially SOD1 and SOD2 [35]. SIRT1 directly deacetylates FOXO1, thereby stimulating the expression of genes that mediate cytoprotective cells [36]. p53 is a transcription factor with a powerful proapoptotic effect and is the first nonhistone deacetylation target of SIRT1. The deacetylation of p53 by SIRT1 is related to the decline of p53 transcription function, thereby inhibiting apoptosis [37]. The activation of NF-*κ*B participates in the occurrence and development of sepsis by enhancing the transcription of various proinflammatory cytokines, including TNF-*α*, IL-6, and IL-1*β*. SIRT1 can deacetylate NF-*κ*B and inhibit the activity of NF-*κ*B, thereby exerting a neuroprotective effect [38]. It can be seen from this study that YBTF downregulated the expression of Ac-FOXO1, Ac-NF-*κ*B, and Ac-p53 in septic mice, thereby confirming that YBTF affects the expression of Ac-FOXO1, Ac-NF-*κ*B, and Ac-p53 by activating the expression of SIRT1 to regulate cognitive dysfunction in septic mice. Meanwhile, it can also enhance the intervention effect of the drug dexamethasone on sepsis in mice by regulating the expression of SIRT1 (Figure 6).

Nine compounds, including catechin, gallocatechin gallate, rutin, hyperoside, epicatechin gallate, dihydroquercetin, quercetin, myricetin, and sulphuretin, have antioxidant and anti-inflammatory effects [39–47]. The combined effect of catechin and epicatechin gallate can effectively inhibit sepsis [48]. Epigallocatechin gallate can regulate the TLR4/Myd88/NF-*κ*B pathway to play a role in septic rats [49]. Myricetin has a protective effect on septic cardiomyopathy in mice [50]. In particular, studies have shown that catechin, rutin, hyperoside, quercetin, and myricetin have certain inhibitory and intervention effects on sepsis [51–54]. This study also showed that YBTF can interfere with sepsis through the action of these 9 active ingredients (Figure 7). The combined effects of these compounds with anti-inflammatory and sepsis inhibition became the key to the action of YBTF in this study.

## 5. Conclusions

In summary, YBTF enhances the survival rate of septic mice by activating SIRT1, increases the activity exploration ability and learning cognitive ability of septic mice, and reduces the rate of neuronal apoptosis, as well as reducing inflammation and oxidative stress. This phenomenon is closely related to the expression of FOXO1, NF-*κ*B, and p53. Meanwhile, YBTF also has the effect of enhancing the efficacy of dexamethasone. These experimental results provide reference data for the treatment of cognitive dysfunction in sepsis, but the exact mechanism governing the effects of TBTF still warrants further investigation. At the same time, YBTF is a complex mixture. In this study, the main compounds were analysed by HPLC, but the compounds need to be comprehensively analysed by liquid chromatography-mass spectrometry.

## Figures and Tables

**Figure 1:** The survival analysis of mice in different groups.

**Figure 2:** The total distance travelled, number of standing episodes, number of self-grooming episodes, time in the target quadrant, and number of times to cross the area of mice in different groups (*n* = 6). Measured value means mean ± SEM value. ^a–e^Mean values with different letters over the bar are significantly different (*P* < 0.05) according to Tukey's honestly significant difference.

**Figure 3:** Apoptosis of nerve cell of septic mice. ^a–d^Mean values with different letters over the bar are significantly different (*P* < 0.05) according to Tukey's honestly significant difference. (a) Normal. (b) Model. (c) Dexamethasone. (d) YBTF. (e) YBTF + dexamethasone.

**Figure 4:** TNF-*α*, IL-6, and IL-1*β* cytokines levels of hippocampus of mice (*n* = 6). Measured value means mean ± SEM value. ^a–e^Mean values with different letters over the bar are significantly different (*P* < 0.05) according to Tukey's honestly significant difference.

**Figure 5:** SOD, CAT, and MDA levels of hippocampus of mice (*n* = 6). Measured value means mean ± SEM value. ^a–e^Mean values with different letters over the bar are significantly different (*P* < 0.05) according to Tukey's honestly significant difference.

**Figure 6:** SOD1, SOD2, CAT, MDA, TNF-*α*, IL-1*β*, NF-*κ*B, p53, FOXO1, and SIRT1 mRNA expression of hippocampus of mice (*n* = 3). Measured value means mean ± SEM value. ^a–e^Mean values with different letters over the bar are significantly different (*P* < 0.05) according to Tukey's honestly significant difference.

**Figure 7:** Constituents of Yunnan black tea flavonoids. (a) Standard chromatograms. (b) Yunnan black tea flavonoids chromatograms. 1, catechin; 2, gallocatechin gallate; 3, rutin; 4, hyperoside; 5, epicatechin gallate; 6, dihydroquercetin; 7, quercetin; 8, myricetin; 9, sulphuretin.

**Table 1:** Sequences of primers used in the qPCR assay.

Gene name	Sequence
SOD1 (Cu/Zn-SOD)	Forward: 5′-AACCAGTTGTGTTGTCAGGAC-3′
	Reverse: 5′-CCACCATGTTTCTTAGAGTGAGG-3′

SOD2 (Mn-SOD)	Forward: 5′-CAGACCTGCCTTACGACTATGG-3′
	Reverse: 5′-CTCGGTGGCGTTGAGATTGTT-3′

CAT	Forward: 5′-GGAGGCGGGAACCCAATAG-3′
	Reverse: 5′-GTGTGCCATCTCGTCAGTGAA-3′

TNF-*α*	Forward: 5′-CACGCTCTTCTGTCTACTGAAC-3′
	Reverse: 5′-ATCTGAGTGTGAGGGTCTGG-3′

IL-1*β*	Forward: 5′-GCAACTGTTCCTGAACTCAACT-3′
	Reverse: 5′-ATCTTTTGGGGTCCGTCAACT-3′

NF-*κ*B	Forward: 5′-CATGTCTCACTCCACAGCT-3′
	Reverse: 5′-CCGGAGAGACCATTGGGA-3′

p53	Forward: 5′-TAACAGTTCCTGCATGGGCGGC-3′
	Reverse: 5′-AGGACAGGCACAAACACGCACC-3′

FOXO1	Forward: 5′-GCACAGTGAACTCCAGGAAAGG-3′
	Reverse: 5′-CACCAAAGGAAATGAATCAAACAAG-3′

SIRT1	Forward: 5′-CAGTGTCATGGTTCCTTGC-3′
	Reverse: 5′-CACCGAGGAACTACCTGAT-3′

GAPDH	Forward: 5′-AGGTCGGTGTGAACGGATTTG-3′
	Reverse: 5′-GGGGTCGTTGATGGCAACA-3′

## Data Availability

The datasets used to support the findings of this study are available from the corresponding author upon request.
